# Analysis of Development Mechanism of Giant Cell Arteritis in Nude Mouse Model through Color Duplex Sonography and Computerized Tomography Nanocontrast Agent

This article has been retracted.

**DOI:** 10.1155/2021/6627925

**Published:** 2021-04-09

**Authors:** Fugang Chen, Yang Li, Hongyan Zhou, Chuang Sun, Sun Li, Lu Wang, Xin Li, Xiaoqiang Liu

**Affiliations:** ^1^Department of Radiology, The Second Affiliated Hospital of Dalian Medical University, Dalian 116031, China; ^2^Department of Ultrasound, The Second Affiliated Hospital of Dalian Medical University, Dalian 116031, China; ^3^Department of Nursing, The Second Affiliated Hospital of Dalian Medical University, Dalian 116031, China

## Abstract

To explore the application value of color duplex sonography and enhanced computerized tomography (CT) inspection based on a nanocontrast agent in diagnosis and pathogenesis in giant cell arteritis (GCA), the GCA nude mouse model was constructed. In this study, 40 healthy male BalB/c nude mice aged 6-8 weeks were randomly divided into a control group (no model) and an experimental group (model), with 20 mice in each group, and the temporal artery tissue of GCA patients diagnosed as positive by temporal artery biopsy was implanted into nude mice to construct a GCA nude mouse model. Abdominal aortic biopsy and immunohistochemistry were used to verify the success of the GCA nude mouse model. All nude mice were subjected to color duplex sonography and enhanced CT examination based on a nanocontrast agent. At the same time, the basic indicators such as body weight, temperature, white blood cell (WBC), lymphocytes (LYM), hemoglobin (HGB), and platelet (PLT) were measured, and the protein expression levels of interleukin-6 (IL-6) and signal transducer and activator of transcription 3 (STAT3) were detected by immunohistochemistry. The results showed that the temporal artery wall of the nude mice in the experimental group thickened and the lumen was significantly narrowed, indicating that the cell arteritis model of nude mice was successfully constructed; ultrasound examination showed that the right superficial temporal artery vascular cavity narrowed, the blood flow signal changed like a filling defect around the periphery, and there was a low echo halo. CT examination showed that the left superficial temporal artery narrowed, and the inner diameter of the narrow segment of blood vessels changed like a bead. The body weight of nude mice in the experimental group decreased significantly after the modeling was completed (*P* < 0.05); after modeling, the body temperature of the nude mice in the experimental group increased significantly (*P* < 0.05); LYM and HGB values of nude mice in the experimental group were significantly lower than those in the control group (*P* < 0.05); the content of IL-6, STAT3, IL-6, and STAT3 proteins in the arterial tissue of nude mice in the experimental group was lower than that of the control group (*P* < 0.05), indicating that color duplex sonography and CT contrast agent technology can be used in the diagnosis and development mechanism research of GC.

## 1. Introduction

GCA is a common large and medium vasculitis, and it is a granulomatous vascular disease that mainly violates the extracranial branches of the aorta such as the ocular artery, superficial temporal artery, vertebral artery, and middle artery. GCA is prevalent in the elderly population over 50 years old in western countries. In recent years, the detection rate of GCA in China has also been increasing [1]. CT imaging technology is widely used in clinical diagnosis because of its strong tissue penetration, low cost, high resolution, and powerful image postprocessing technology. Common CT scanning methods in clinic include routine scanning and enhanced scanning. Among them, the enhanced scan introduces a contrast agent into the body to enhance the contrast of the observed object, and it is easy to distinguish the lesion area [2]. CT contrast agents currently used clinically are mainly iodine contrast agents; however, large doses of iodine can cause harm to the human body. At the same time, the process of kidney removal of iodine molecules will affect angiography and imaging [3]. A nanocontrast agent has the characteristics of high contrast, long cycle time, and higher X-ray attenuation coefficient than iodine. It has attracted extensive attention from researchers in various fields. At present, CT contrast agents have been widely used in the examination and diagnosis of the head and neck, chest, liver, lung, kidney, spleen, abdominal aorta, bladder, and other parts of the body [4].

Commonly used methods for clinical diagnosis of GCA include angiography, computerized tomography angiography (CTA), magnetic resonance angiography (MRA), and dual-function color ultrasound. Among them, angiography is the gold standard for the diagnosis of vascular diseases; however, in the course of clinical use, it is not only expensive, but also traumatic and prone to complications [5]. The examination of small blood vessel lesions by MRA is limited by the spatial resolution, and the imaging of narrow blood vessels will exaggerate the lesions [6]. Color duplex ultrasound technology can determine the best location of the superficial temporal artery biopsy. It is widely used in the diagnosis and treatment of heart diseases because of its low cost, simple operation, and strong repeatability. It is also considered to be the preferred method for the diagnosis of GCA, but its sensitivity to detect arterial walls is not high [7], which needs to be used in combination with other diagnostic methods.

At present, the etiology and pathogenesis of GCA are still unclear. Due to limitations of experimental techniques and diagnostic conditions, most of the current research on GCA uses clinical collection of patient data for retrospective analysis. There are great limitations due to uncontrollable factors that interfere with the data collection process. Therefore, using animal models to study the mechanisms of occurrence and development of GCA has significant advantages, and has important significance for the study of the etiology and pathogenesis of GCA. However, there are few reports on GCA modeling, and there are problems such as difficulty in modeling technology and poor repeatability.

This study was based on the fact that there is no mature and reliable GCA animal model. Combined with the advantages of color duplex sonography and CT nanocontrast agent, 6–8-week-old healthy male BalB/c nude mice were used as the research object to transplant the temporal artery of GCA patients to nude mouse abdominal aorta, to simulate the pathophysiological environment of the disease in the human body as much as possible. A nude mouse GCA model was established, and through color duplex sonography and CT nanocontrast agent analysis of the model, the occurrence and development mechanism of nude mouse GCA was explored, to provide a reference for clinical diagnosis and treatment of GCA.

## 2. Materials and Methods

### 2.1. Test Animals and Materials

Forty 6–8-week old healthy male BalB/c nude mice, weighing 18-23 g, were kept in a clean laboratory animal room, with a room temperature of 25°C, a relative humidity of about 55%, and under 12 hours of light. They were free to drink water and eat. After 2 weeks of adaptive feeding of all mice, all nude mice were randomly divided into a control group and an experimental group, with 20 mice in each group. The nude mice in the experimental group were modeled, while the control group was not. All nude mice were fasted for 12 hours before modeling. The 2-4 segments of the temporal artery tissue of GCA patients diagnosed as positive by temporal artery biopsy were implanted into BalB/c nude mice. Temporal artery biopsy and monocyte isolation of GCA patients involved in this trial were all approved by the ethics review committee of the Second Affiliated Hospital of Dalian Medical University, and all patients or their legal representatives had signed the informed consent. All animal procedures were approved by the Experimental Animal Management Committee, and the experimental methods were carried out in accordance with the approved guidelines.

### 2.2. Establishment of GCA Nude Mouse Model

The nude mice were placed in a sterile operating table and anesthetized with l% pentobarbital sodium. After anaesthesia, the skin preparation was performed and a longitudinal opening in the center of the abdomen was carried out to fully expose the anterior abdominal wall. A cotton swab was used to pick out the intestine and place it on the gauze infiltrated with warm saline to expose the abdominal artery by about 1.5 cm. Noninvasive microvascular clips were used to clamp the abdominal main branch of the renal artery branch about 0.3 cm and 1.2 cm down the artery. In the operation, an incision with a size of 0.1 cm × 0.3 cm was cut between the two invasive microvascular clips, the incision was rinsed with a small amount of prewarmed physiological saline, and the temporal artery tissue of GCA patients with the size of the incision was implanted. A no. 11-0 suture was performed, and the vascular clamp was removed to observe the pulsation regularity of the aorta. After the success of the implantation operation, the intestinal canal was carefully placed in the nude mouse body, and the peritoneal muscle layer and the skin layer were sutured with layered sutures using a no. 5-0 suture. After successful modeling, all nude mice were placed in cages, reared normally, and were free to drink water. One month later, all nude mice were killed, and the abdominal aorta specimens of nude mice were collected.

### 2.3. GCA Nude Mouse Model Identification

The hematoxylin-eosin (HE) staining method was used to observe the morphology of the abdominal aorta in the nude mice in the control group and the GCA model nude mice; under the electron microscope, the maximum intima and media thickness of the abdominal aorta in mice was observed. Immunohistochemical staining was used to analyze the temporal artery tissues of nude mice in control nude mice and GCA model nude mice.

### 2.4. Enhanced CT Scan

Enhanced CT scans were performed on all nude mice the day before sacrifice. The hydrothermal method was used for preparation of monodisperse nanoparticles Yb(OH)CO_3_ [8], and the in vitro hemolysis analysis method [9] was used for verification of nanoparticle Yb(OH)CO_3_. Then, it was used as a contrast agent, and all nude mice were injected with 1 mL Yb(OH)CO_3_ solution with a concentration of 50 mg/mL. A Philips 256-slice spiral CT was used for scanning. The scanning voltage was 120 kV, the scanning current was 300 mA, the layer thickness was 0.9 mm, and the pitch was 0.99. The tube rotation time was 0.5 s. All original images obtained by CT scanning were transferred to the Wizard workstation for image postprocessing.

### 2.5. Inspection Method of Color Duplex Sonography in Nude Mice

Nude mice were examined using the GE Vivid 17 and GE Vivid 7 Dimension color Doppler ultrasound system. The probe was a high-frequency linear array probe, and the probe frequency conversion range was 7.0-11.4 Hz. During the examination of the superficial temporal artery and branch vessels, the focus point should be placed as close to the field as possible to fully expose the bilateral temporal part. A two-dimensional ultrasound examination of the parietal and frontal branches was performed to observe the superficial temporal artery and branch vessels and the ultrasonic anatomy of the vessels.

### 2.6. Method of Detecting Basic Indicators of Nude Mice

The body temperature and body weight of two groups of nude mice were detected, and the changes of body temperature and body weight of the two groups of nude mice were recorded and compared before and after modeling, 1 week after modeling, 2 weeks after modeling, 3 weeks after modeling, and before sacrifice. The detection method of anal temperature referred to the research of Asamoah and Ansah-Mensah in 2020 [10]. Before testing, animals were allowed to empty their stools, and the anal temperature of all nude mice was recorded. The anal temperatures of two groups of nude mice before modeling, at the end of modeling surgery, 1 week after modeling, 2 weeks after modeling, 3 weeks after modeling, and before sacrifice were recorded, and the changes of body temperature of mice in each group at each time point were calculated. Before the nude mice were killed, 0.5 mL of whole blood was taken from the orbital venous plexus in EDTA K2 anticoagulation tubes and 1.5 mL centrifuge tubes, and the centrifuge tubes were spun in centrifuge at 3000 r/min for 10 minutes. An automatic blood cell analyzer was used to detect the whole blood routine indicators of all nude mice, including WBC, LYM, HGB, and PLT.

### 2.7. Detection of IL-6 and STAT3 Protein Expression Levels

The immunohistochemical method was used to detect the protein expression levels of IL-6 and STAT3 proteins. The primary antibodies against IL-6 and STAT3 were used to perform conventional immunohistochemistry to observe tissue staining under the microscope. The IL-6-positive cells were microscopic brown particles in the cytoplasm under a microscope. The positive standard of STAT3 was that the cytoplasm was stained brown. The analysis software Image-Pro Plus 6.0 was used to determine the average optical density of the positive cells.

### 2.8. Statistical Analysis

SPSS 19.0 was used for data statistics and analysis. Measurement data were expressed as mean ± standard deviation ($\bar{x}\pm s$). Measurement data that obeyed normal distribution were tested by *t*-test, and measurement data that were not obeyed normal distribution were tested by Wilcoxon test. One-way analysis of variance was used for comparison. *P* < 0.05 was statistically significant.

## 3. Results

### 3.1. Results of Analysis of CT Nanocontrast Agent Detection In Vitro

The hemolysis of the nanocontrast agent was detected at a wavelength of 541 nm. The nanocontrast agent and PBS did not experience hemolysis, indicating that the nanoparticles had good blood compatibility, which provided feasibility for further studies in vivo. The results are shown in Figure 1.

### 3.2. GCA Nude Mouse Model Verification

The abdominal aortas of the nude mice in the control group and the GCA model were observed by the HE staining method, and the results are shown in Figure 2. The abdominal aorta thickness of the nude mice in the experimental group (Figure 2(a)) was significantly higher than that of the control group (Figure 2(b)) (arrows in the figure). It can be found from the immunohistochemical images of the temporal arteries of the nude mice of the control group and the GCA model that compared with the control group (Figure 2(d)), the temporal artery wall of the experimental group of nude mice thickened and the lumen was significantly narrowed. From the perspective of mononuclear cell infiltration, there was much mononuclear cell infiltration in the temporal artery of nude mice in the experimental group, and the full-thickness cracking phenomenon of blood vessels appeared.

### 3.3. Results of Analysis of Color Duplex Sonography Scan of Nude Mice

Color duplex sonography scan was performed in nude mice in the control group and the experimental group, and the results are shown in Figure 3. Compared with the control group (Figure 3(a)), the wall of the left superficial temporal artery main vessel of nude mice in the experimental group (Figure 3(b)) was thickened concentrically, the echo was reduced, the inner diameter of the vascular cavity was narrowed, and the blood flow showed a local continuous interruption. Compared with the control group of nude mice (Figure 3(c)), the right superficial temporal artery trunk cavity of nude mice in the experimental group (Figure 2(d)) narrowed, the blood flow signal changed like a peripheral filling defect, and there was a low echo halo. The left branch of the superficial temporal artery of nude mice in the experimental group was filled with solid hypoechoic luminous clusters, and the blood vessel wall thickened (Figure 3(e)). At the same time, it can be found that the diameter of the left lumen of the superficial temporal artery of the nude mice in the experimental group narrowed, the blood vessel wall thickened, and the echo increased (Figure 3(f)).

### 3.4. Results of Analysis of GCA Model Nude Mice Using Enhanced CT Scan

The GCT model of nude mice in the experimental group was subjected to enhanced CT scan. The results are shown in Figure 4. The left superficial temporal artery narrowed, and the inner diameter of the narrow segment of the blood vessel changed like a bead (Figure 4(a)). The right branch of the artery showed a segmental narrowing, and the lumen of the vessel was irregularly narrowed (Figure 4(b)).

### 3.5. Weight Change Analysis of GCA Model Nude Mice

The weights of two groups of nude mice before and after modeling were tested. The results are shown in Figure 5. The weights of the nude mice in the control group and the experimental group before modeling were 19.74 ± 1.43 g and 19.53 ± 1.78 g; there was no significant difference in body weight between the two groups of nude mice (*P* > 0.05). At the same time, there was no significant difference in body weight between the two groups of nude mice at the end of the modeling operation and within 1 week after modeling. After 2 weeks of modeling, the body weight of the two groups of nude mice was detected, and it was found that the weight of the nude mice in the experimental group obviously decreased. Compared with the body weight of the control nude mice in the same period, there was a significant difference (*P* < 0.05); from 2 weeks after modeling, with the extension of time, the weight loss of nude mice in the experimental group was more obvious, and there was a significant difference compared with the control group (*P* < 0.05), and there was no significant difference between the weight before sacrifice and the weight at the beginning of the experiment (*P* > 0.05). Throughout the experimental period, the weight of nude mice in the control group continued to rise, and there was a very significant difference between the weight before sacrifice and the weight at the beginning of the experiment (*P* < 0.01).

### 3.6. Analysis of Anal Temperature Changes of GCA Nude Mice

The body weight of the two groups of nude mice before and after modeling was tested. The results are shown in Figure 6. The anal temperature of the control group of nude mice was basically stable during the entire experiment period. The anal temperature of nude mice before the experiment and before modeling was not different from that of the control group (*P* > 0.05). From the first week after surgery, the temperature of the nude mice in the experimental group showed an upward trend. Compared with the control group, the anal temperature increased by 0.97 ± 0.26°C, and the difference was statistically significant (*P* < 0.05). Compared with the average anal temperature before the experiment started, the average anal temperature of the nude mice in the experimental group before sacrifice increased by 0.92 ± 0.19°C, and the difference was statistically significant (*P* < 0.05).

### 3.7. Analysis of Biochemical Indexes of Two Groups of Nude Mice

The WBC, LYM, HGB, and PLT of the two groups of nude mice were tested and analyzed. The results are shown in Figure 7. The WBC and PLT values of nude mice in the control group were not significantly different from the experimental group (*P* > 0.05). The LYM and HGB values of nude mice in the control group were higher than those in the experimental group, and they were statistically significant compared to the experimental group (*P* < 0.05).

### 3.8. IL-6 and STAT3 Protein Expression Level Detection

The immunohistochemical method was used to stain the IL-6 and STAT3 proteins in the arterial tissues of the nude mice in the experimental group and the control group. The results are shown in Figure 8. IL-6 protein and STAT3 protein expression staining were all in the cytoplasm and widely distributed in the intima, media, and adventitia of blood vessels. At the same time, it can be found that the nude mice in the control group had cell infiltration. The IL-6 and STAT3 protein contents in the arterial tissues of the two groups of nude mice were measured and compared. The results are shown in Figure 9.

The IL-6 and STAT3 protein contents in the arterial tissues of nude mice in the experimental group were 3.93 ± 0.4 and 41.59 ± 2.25, respectively. The IL-6 and STAT3 protein contents in the arterial tissue of nude mice in the control group were 2.16 ± 0.51 and 29.87 ± 2.84, respectively. The IL-6 and STAT3 protein levels in the arterial tissues of nude mice in the control group were lower than those in the experimental group, and the difference was statistically significant (*P* < 0.05).

## 4. Discussion

In this study, color duplex sonography and enhanced CT scanning with a nanomolecular contrast agent were used to find out the imaging characteristics of the superficial temporal artery of GCA nude mice, and the development mechanism of GCA was discussed in combination with biochemical indexes, basic indexes, and vascular tissue biopsy results. GCA lesions involve the large and middle arteries of the whole body, so the use of traditional modeling methods has great limitations [11]. In this study, the temporal artery tissue of GCA patients was implanted into the anterior wall of the aorta of healthy male BalB/c nude mice. A GCA animal model was established. The abdominal aorta was morphologically observed and identified by immunohistochemical staining. The thickness of the aorta was significantly higher than that of the control group, the wall of the temporal artery was thickened, the lumen was significantly narrowed, there was much mononuclear cell infiltration in the temporal artery, and the phenomenon of a full-thickness crack appeared. These characteristics indicated that the nude mice in the experimental group showed symptoms of inflammatory damage and increased inflammatory cells, which was consistent with the current results of GCA biopsy [12], which fully illustrated the success of the construction of the GCA animal model in this study. The clinical diagnosis of superficial temporal artery GCA mainly depends on arterial angiography and biopsy [13]. With the rapid development of multilayer high-speed spiral CT scanning technology, color duplex sonography and enhanced CT examination have become the preferred examination methods for observing changes in the superficial temporal artery [14]. In this study, two groups of nude mice were subjected to color double ultrasound and enhanced CT examination. During the enhanced CT examination, nanoparticles were used as contrast agents to increase the contrast and resolution of the image. Color duplex sonography examination found that the left superficial temporal artery main vessel wall of the nude mice in the experimental group was thickened concentrically, the echo was reduced, the inner diameter of the vascular cavity was narrowed, and the blood flow showed local continuous interruption; the vascular lumen of the main trunk of the right superficial temporal artery was narrowed, and the blood flow signal showed a peripheral filling defect with a hypoechoic halo. A large number of studies have shown that the right superficial temporal artery main artery presents blood flow signal changes like a peripheral filling defect and has a hypoecho halo, which is the characteristic image of superficial temporal artery GCA [15]. Studies have found that ultrasound of GCA shows irregular thickening of arterial vascular intima, mild stenosis of blood vessel lumen, clear boundary between diseased vessels and surrounding tissues, irregular thickening of arterial vascular intima, and enhanced echo [16]. The ultrasound examination results in this study were consistent with the GCA ultrasound features reported so far. In this study, the enhanced CT examination of the GCA model nude mice found that the superficial temporal arteries of the nude mice were narrowed, the inner diameter of the narrowed blood vessels changed like a bead, and the vascular cavity was irregularly narrowed. In 2019, Bley and Dechant [17] performed CTA examination on GCA patients, and it was found that the inner diameter of the vascular cavity of the superficial temporal artery lesion was irregularly narrowed, which was consistent with the results of the enhanced CT examination in this study.

In this study, the basic data and biochemical indicators of the two groups of nude mice were tested and analyzed at the same time. The results showed that the body weight of the nude mice in the experimental group decreased significantly after the modeling was completed (*P* < 0.05). Compared with the control group of nude mice (*P* < 0.05), GCA nude mice had symptoms of weight loss and body temperature increase, which was consistent with the symptoms of GCA patients of the previous foreign and domestic studies [18]. At the same time, it was found that the LYM and HGB values of the nude mice in the control group were higher than those in the experimental group (*P* < 0.05), which was consistent with the current biochemical index test results of GCA patients. The levels of IL-6 and STAT3 protein in nude mice in the experimental group were higher than those in the control group. In 2019, Weyand et al. [19] proposed that immune factors participated in the pathogenesis of arteritis, and the expression level of IL-6 increased, which was a typical feature of GCA patients. The persistent symptoms of patients were closely related to the increase of IL-6 expression levels [20].

## 5. Conclusion

By establishing a GCA nude mouse model, the characteristics of GCA color duplex sonography and enhanced CT scan images using nanosmall molecules as contrast agents were explored. Combining biochemical indicators and vascular tissue biopsy results, the development mechanism of GCA was discussed. The results showed that the GCA implantation method was successfully used to construct the nude mouse model. The results of color duplex sonography and enhanced CT using small nanomolecules as contrast agents were consistent with clinical biochemical indicators and vascular tissue biopsy results, indicating that color duplex sonography and CT contrast agent technology can be used in the diagnosis of GCA. However, there were still some shortcomings in this study. This study mainly analyzed the changes of the superficial temporal artery, but did not analyze the structural changes of other arteries. In the subsequent research, other large and middle arteries should be analyzed. In conclusion, color duplex sonography and CT contrast agent technology can be used in the diagnosis and development mechanism research of GCA.

## Figures and Tables

**Figure 1:** CT nanocontrast agent hemolytic result analysis.

**Figure 2:** GCA nude mouse model verification: (a) HE staining figure of the abdominal aorta in mice from the experimental group; (b) HE staining figure of the abdominal aorta in mice from the control group; (c) temporal artery immunohistochemistry figure of nude mice from the experimental group; (d) temporal artery immunohistochemistry figure of nude mice from the control group.

**Figure 3:** Color duplex sonography scan image of nude mice. (a) Color duplex sonography scan image of the left superficial temporal artery main vessel of nude mice from the control group. LMSTA: left superficial main vessel temporal artery. (b) Color duplex sonography scan image of the left superficial temporal artery main vessel of nude mice from the experimental group. LMSTA: left superficial main vessel temporal artery. (c) Color duplex sonography scan image of the right superficial temporal artery main artery of nude mice from the control group. RMSTA: right main superficial temporal artery. (d) Color duplex sonography scan image of the right superficial temporal artery main artery of nude mice from the experimental group. RMSTA: right main superficial temporal artery. (e) Color duplex sonography scan image of the left branch of the superficial temporal artery of nude mice from the experimental group. LTB: left branch of the temporal artery. (f) Color duplex sonography scan image of the right branch of the superficial temporal artery of nude mice from the experimental group. RTB: right temporal artery branch.

**Figure 4:** GCA model of nude mouse subject to enhanced CT scan. (a) Enhanced CT scan image of the left branch of the superficial temporal artery in GCA model of nude mice. LTB: left branch of the superficial temporal artery. (b) Enhanced CT scan image of the right branch of the superficial temporal artery in GCA model of nude mice. RTB: superficial temporal artery right branch.

**Figure 5:** Comparison of body weight between two groups of nude mice at different time periods (∗ indicates a notable difference versus the control group, *P* < 0.05; # indicates a notably significant difference versus the test group, *P* < 0.01).

**Figure 6:** Comparison of anal temperature between two groups of nude mice at different time periods (∗ indicates a notable difference versus the control group, *P* < 0.05; # indicates a notable difference versus the test group at the beginning, *P* < 0.05).

**Figure 7:** Comparison of biochemical indexes of two groups of nude mice (∗ indicates a notable difference versus the control group, *P* < 0.05).

**Figure 8:** IL-6 and STAT3 protein expression staining results in nude mouse arterial tissue: (a) IL-6 protein expression in the arterial tissue of nude mice in the control group; (b) STAT3 protein expression in the arterial tissue of nude mice in the control group; (c) IL-6 protein expression in the arterial tissue of nude mice in the experimental group; (d) STAT3 protein expression in the arterial tissue of nude mice in the experimental group.

**Figure 9:** Comparison of IL-6 and STAT3 protein expression in arterial tissues of two groups of nude mice (∗ indicates a significant difference compared with the control group, *P* < 0.05).

## Data Availability

Some or all data, models, or code generated or used during the study are available from the corresponding author by request.
